The article "Risk and causality Co-movement of Malaysia’s stock market with its emerging and OECD trading partners. Evidence from the wavelet approach" was retracted in 2025. Reasons: unreliable results or conclusions; concerns about the peer review; concerns about the authorship.

# Risk and causality Co-movement of Malaysia’s stock market with its emerging and OECD trading partners. Evidence from the wavelet approach

**DOI:** 10.1371/journal.pone.0296712

**Published:** 2024-01-25

**Authors:** Xiaoyang Wang, Hui Guo, Muhammad Waris, Badariah Haji Din

**Affiliations:** 1 Innovation College, North Chiang Mai University, Nong Kaew, Hong Dong, Chiang Mai, Thailand; 2 Xuchang Industrall & Commerclal Administration School No.3, Jian’an District, Xuchang City, Henan Province, China; 3 Ghazali Shafie Graduate School of Government, University Uttara Malaysia, Malaysia, Malaysia; University of Southampton - Malaysia Campus, MALAYSIA

## Abstract

The growing trend of interdependence between the international stock markets indicated the amalgamation of risk across borders that plays a significant role in portfolio diversification by selecting different assets from the financial markets and is also helpful for making extensive economic policy for the economies. By applying different methodologies, this study undertakes the volatility analysis of the emerging and OECD economies and analyzes the co-movement pattern between them. Moreover, with that motive, using the wavelet approach, we provide strong evidence of the short and long-run risk transfer over different time domains from Malaysia to its trading partners. Our findings show that during the Asian financial crisis (1997–98), Malaysia had short- and long-term relationships with China, Germany, Japan, Singapore, the UK, and Indonesia due to both high and low-frequency domains. Meanwhile, after the Global financial crisis (2008–09), it is being observed that Malaysia has long-term and short-term synchronization with emerging (China, India, Indonesia), OECD (Germany, France, USA, UK, Japan, Singapore) stock markets but Pakistan has the low level of co-movement with Malaysian stock market during the global financial crisis (2008–09). Moreover, it is being seen that Malaysia has short-term at both high and low-frequency co-movement with all the emerging and OECD economies except Japan, Singapore, and Indonesia during the COVID-19 period (2020–21). Japan, Singapore, and Indonesia have long-term synchronization relationships with the Malaysian stock market at high and low frequencies during COVID-19. While in a leading-lagging relationship, Malaysia’s stock market risk has both leading and lagging behavior with its trading partners’ stock market risk in the selected period; this behavior changes based on the different trade and investment flow factors. Moreover, DCC-GARCH findings shows that Malaysian market has both short term and long-term synchronization with trading partners except USA. Conspicuously, the integration pattern seems that the cooperation development between stock markets matters rather than the regional proximity in driving the cointegration. The study findings have significant implications for investors, governments, and policymakers around the globe.

## 1. Introduction

The stock market is an integral part of each economy that leads to economic growth and industrial development within the nation. Stock markets fulfill the financial needs of the corporate sector and may open different opportunities for investors to earn profit from trading in the stock market. Many aspects, such as crises, pandemics, and environmental changes, affect the stock market. The fluctuation in the stock market prices creates a risk for investors. Still, due to globalization, the risk transfer from one economy to another makes this task worse for the investors of the international portfolio. Globalization has strengthened the linkage between international stock markets. Through globalization, cross-border trade is boosted by eliminating the barriers to stock market integration [1, 2]. Therefore, with the stock market fluctuation, the risk and causality transmission create another problem for the investors.

Similarly, the stock market of Malaysia shows different patterns in pre- and post-crisis. However, the crisis and the pandemic affected the pattern of the Malaysian stock market, creating different economic challenges. The Asian Financial Crisis 1997 98 is considered one of Malaysia’s most crucial economic crises. This crisis created the deregulation of the capital accounts and the financial sector, which caused a decline in the GDP growth of 6.7% or 7.7% before the crisis period. This crisis on the first day decreased the Kula lumper stock exchange to 44.9%. The value of the currency ringgit also fell in January 1998. There is enormous pressure on both the currency and financial markets due to the crisis. In the financial crisis of 2008–9, there was a decline in the total GDP to 1.7% in 2009 and had some other negative consequences.

Moreover, due to COVID-19, all financial activities have dropped in the world, including the downsizing in the stock market prices. Like the other economy, Malaysia was also affected by the country’s lockdown. According to [3], Malaysia’s stock market indices have dropped and are highly correlated with the pandemic.

Moreover, the crisis in one economy affects the other stock market because a correlation exists between them due to globalization that creates another issue. Similarly, When the Malaysian market is affected by the crashes, it may impact the trading partners in different world regions. When the Stock market of Malaysia (Kula Lumpur Stock Exchange) declined due to the crisis in 2008, it also decreased in the Japanese stock exchange due to the significant foreign direct investment made by Japan in Malaysia. The Chinese stock market crash of 2015 affected the Malaysian stock market due to the interdependence among the stock markets. At that time, the oil prices also hit Malaysia to its lowest in six years. Gold was considered the safe market during the crisis, but gold prices decreased in China and impacted the Malaysian economy. Moreover, emerging and the OECD economies also effected in the crisis period that are highly independent. Hence, this study mainly investigated the pattern and cointegration between Malaysia, OECD, and emerging countries pre- and post-crisis.

The increased capital flow between countries due to globalization through the rapid development of technology is the cause of the economic integration between different markets and has played an essential role over the last two decades. Every financial institution and portfolio management needs to understand the extent and nature of the linkage between financial markets [4]. The nexus of interdependence between these markets can be analyzed by finding return and volatility transfer between these different financial markets. Risk and causality transmission is crucial for designing hedge strategies and making optimal portfolios. [5] find the emerging markets are severely affected by the different crises in history, and these effects are transmitted to other countries. However, cointegration between the stock market has excellent indicators showing the risk and causality that may transfer from Malaysia to its trading partners in the two regions. Therefore, the main reason behind that factor is the increase in the capital flow among these countries and the rapid development of the technology enhancement between the market that is observed in globalization.

Moreover, the trade volume of Malaysia between emerging and OECD countries grew at different rates in the last 20 years. Therefore, when trade volume between different markets, regions, and countries changes, it also changes the market volatility transmission. Moreover, Malaysian trade with OECD and emerging economies. However, it is essential to investigate the risk and causality transfer from the Malaysian market to its trading partners because of the increasing trend of the trade volume existence that created the interdependence between them over the last two decades. Moreover, each crisis has a different intensity and has different behavior of transfer from one economy to another, such as leading and lagging behavior between markets due to the type of trade and foreign direct investment. Therefore, this study examines the risk and causality transmission between different markets during the major financial crisis (financial crisis in 1997–98, 2008–09, and the period of the pandemic 2020–21).

Various studies have been conducted on the stock market cointegration by focusing on the major economic crisis in the world [6]. In addition to these studies, the International Monetary Fund, Banks for International Settlements, Financial Stability Board (FSB), and other regulatory bodies have examined the connection between global stock markets and systemic risks that were typically undervalued before the crises. These investigations again identified the fragmented local markets as the primary cause of the crises, which led to excessive market volatility and links between the stock market [7]. Most previous research had found substantial levels of linkage among developed markets with few opportunities for diversification. Nevertheless, research on the emerging market is growing to find opportunities for diversification [8]. Moreover, limited studies on the risk transformation in the period of crisis and pandemics, especially in emerging economies such as Malaysia, create an exciting gap for the investigation.

Accordingly, our study aims to investigate the stock market risk co-movement between Malaysia and its trading partners in different time and frequency domains. We aim to answer our research questions about Transferring the risk and causality from the Malaysian stock market to its trading partners pre- and post-crisis. Some motivation points behind our research include it is exciting to focus on Malaysia with its trading partners belonging to emerging and OECD countries as Malaysia is a rapidly growing emerging market with increasing market capitalization and trade partnership with attracting foreign direct investment inwards from different emerging and OECD economies. Malaysia has had a significant role and has become one part of the main engine of the world economy in the last two decades. Malaysia has a substantial role in neighboring countries’ economies and also in all Asian economies.

Similarly, we contributed to the literature in the current study through theoretical, variable, and methodological contributions. First, it contributes fresh evidence of the stock market integration with its emerging and OECD trading partners at different time intervals. Also, it contributes to the literature on co-movement and covariance by exploring the capital markets related to two different regions, including Emerging and OECD countries, that have gained little attention in previous studies. Second, it contributes to the existing theory information that trade agreements and other financial contracts between the economies can provide a hedge and safe opportunity for the investors following the co-integration patterns. Still, the previous theory states that investment in some developed economies like the USA and the UK provides investors with a safe, even opportunity. Third, this research used the stock market indices and employed the three-dimensional wavelet methodology that simultaneously measures the co-movement based on the multiple investment horizons over time.

Moreover, to the best of my knowledge, this research is the first to use the complete wavelet methodology and wavelet based DCC-GARCH for calculating the co-movement of Malaysia with its trading partners belonging to two different regions in both time and frequency domains. In addition, another aspect of this research is the use of wavelet coherency, which is helpful for the investigation. The use of wavelet coherency in this research to examine whether economic and financial considerations justify coherence in co-movement at different time frequencies is also a great feature of the methodology. Fourth, this study contributes to the growing body of literature on the impact of crisis and pandemic by presenting the new data calculated with the help of DCC-GARCH variance to check the influence of the global financial crisis of 1997–98, 2008–9 and the COVID-19 stress on emerging and OECD stock markets. Moreover, this research adds to the literature on the interdependence between Malaysia and the emerging OECD stock market at different investment horizons; there is still little evidence from previous studies on that subset. This research adds to the previous literature by investigating the global stock market uncertainty during the crisis that caused the cointegration fluctuation between the stock markets and also a contribution focused on the financial crisis of 1997–98, 2008–9, and COVID-19 on the short- and long-term dynamic linkage of emerging and OECD capital markets.

The remaining paper is organized as section 2, which discusses the literature review, including the theoretical and empirical literature. The methodology with the data description is included in section 3, and estimated models are explained. The results and their discussion are illustrated in section 4, and the conclusion recommendations with policy implications and limitations are discussed in section 5. Moreover, the future research suggestions are also discussed in section 5.

## 2. Literature review and hypothesis development

The cointegration of the stock markets means the correlation or co-movement between different stock market prices [9–11]. Stock market co-movements have restructured global investment markets, making it a leading research topic. Following groundbreaking work by [6, 12], stock market co-movements have attracted significant research attention by presenting numerous theoretical models that attempt to elucidate the issue further. There is an increasing trend in research on the co-integration of the stock markets due to the effect of the financial crisis. There is an increase in portfolio shock due to the strong integration between the stock markets of different economies, which is a response to the increased integration of the markets. The contagion effect could be felt worldwide, in both emerging and developed markets. This was a direct result of the financial crisis, which resulted in a significant credit crunch due to the collapse of financial markets. Among the events covered in the literature review section are the stock market movements during the devaluation of the Mexican peso in 1994, the East Asian financial crisis in 1997, the global financial crisis in 2009, the Chinese devaluation in 2015, and the period of the pandemic, such events have been the subject of numerous studies, some of which are presented in the literature review section of this study [6, 13]. Apart from such studies, the International Monetary Fund (IMF), the top global economic financial institutions, Banks for International Settlements, the Financial Stability Board (FSB), and other regulatory bodies have examined the relationship between international stock markets and the systemic risks which went generally undervalued before the crises. These investigations consistently pointed to disordered local markets as the initial source of the crises, which resulted in surplus market interconnections and stock market interconnections as a result of interconnections [14, 15]. Previous studies have discovered high levels of interconnection among developed markets, with few opportunities for diversification in most cases. Nonetheless, studies on emerging markets are becoming increasingly popular as investors look for opportunities to diversify their portfolios.

A high degree of interconnection between developed markets has been investigated in most previous studies, with little prospect for diversification. On the other hand, studies on the emerging market are becoming increasingly popular as investors seek diversification opportunities. Various theoretical explanations for stock market linkages have emerged from the growth economies of knowledge on the subject, including the law of one price and theories of stock market movement and stock market interdependence derived from Modern portfolio theory, which all serve to justify stock market linkages [16, 17]. Theories underline portfolio diversification in global markets [18–20]. Prospect theory asserts that investors’ similar expectations about their investments serve as accurate indicators of the performance of their investments. The arbitrage pricing theory, Capital asset pricing theory, assesses the risk principles. It is supported by the principle of interconnectedness of international markets and that asset pricing theory and arbitrage pricing theories depend on a commodity with the same unit price in all international markets.

Similarly, according to the stock market efficiency theory, stock price information flows between international stock markets create a connection between them. According to behavioral finance theory, investor preferences are based on subjective factors that cause herd effects, which cause stock markets to become more correlated. The information spillover effect is analogous to the stock market efficiency theory, which holds that stock market information is the most critical factor in determining the level of correlation between stock markets. It is also assumed that disseminating stock information across countries, regions, and time zones contributes to the correlation between stock information and the performance of international stock markets. Equity market consensus measures are widely regarded as a gold standard for evaluating the benefits of portfolio diversification for investors and the real economy regarding economic growth and global market connectivity, among other things.

[20] state that Malaysia’s stock market indices have dropped and are highly correlated with the pandemic. The global economic crisis is the leading cause of the rise in oil prices, another main economic problem.

[21] explained the different equity markets and found the interconnectedness of the US, UK, and EU markets that played a critical role in strengthening their respective currencies and exchange rates, distinguishing them from other economies. These three markets’ interconnectedness and coordination have fostered their strong financial positions.

Many researchers have studied the past impact of stock market volatility on economic development, but their conclusions have conflicted. Nigeria’s stock market volatility was studied from 1986 to 2010 by [22]. [23] evaluated the relationship between Malaysian stock market volatility and macroeconomic indicators. They found only consumer price index and interest rate volatility Granger substantially affect volatility in stock market returns. Macroeconomic conditions don’t affect the stock market’s performance. Only the money supply volatility has a meaningful link with stock market volatility as per their regression studies.

A considerable study has been undertaken on the impact of domestic stock market cointegration with the global stock market, concentrating on stock market links, integration, and interdependence on an integrated stock market in which marketplaces are linked. After the global financial crisis of 2007–2009, [24] examined six East Asian stock markets and found that the market was less tolerant to shocks from US stock market movements. [25] deeply analyze India’s stock and growing markets.

By applying the different classification systems [26, 27], study the relationship between the ASEAN-5 countries’ stock markets (Indonesia, Singapore, Malaysia, Thailand, and the Philippines) and the world’s developed stock markets (the United States stock market and the Asian stock market such as Japanese Stock Market) and concluded that cointegration between ASEAN-5 stock prices, US stock prices, and Japanese stock prices persists through time, with a stronger cointegration during crisis period. Consequently, emerging stock markets are especially vulnerable to changes in the stock markets of developed countries, particularly in the United States of America (USA). The stock markets of the ASEAN-5 countries are closely linked to those of the United States and Japan, and this linkage was solid before the financial crisis. Their findings also show that emerging stock markets are highly vulnerable to the volatility of stock markets in developed countries, particularly the United States. As a result of [28] research on four international stock exchanges (the U.S., the ASEAN block, Asia, and the world), the national and international stock exchanges have a variety of channel connections. However, there was a clear link between domestic and international markets regarding integration. [29] examined Asian capital market cointegration and found opportunities for diversification to potential investors in Pakistan, India, Bangladesh, and China, respectively.

More research has been conducted to investigate the reasons for stock market volatility, including macroeconomic factors. [28]) conducts a series of tests based on long-term monthly data for the United States to discover the macroeconomic factors for stock market fluctuations. [30–33] provide additional data on the macroeconomic determinants of market volatility. As a result of the interdependence of markets, there are three possible paths: shared shocks, trade ties with competitive devaluations, and financial links. There is a wide range of market connections that have contributed to the establishment of these channels. As an example [34], cite significant increases in global or US interest rates [35], lists changes in commodity prices as well as recessions in major industrial countries, and [36] includes slowdowns in US or global industrial production as well as changes in the ratings of developed countries.

Moreover [37], argue that the developed market of the United States has a more significant effect on the Australian stock market than other countries in the region, but this is not true for the other Pacific Basin countries. This study examined the relationship between the stock markets of Pacific Basin nations from 1988 to 1996. Moreover [38], investigated the region of Scandinavian countries and the United States of America during the same period to see whether US stock transactions had an impact on the countries and found the high co-integration between these economies.

[39] found little correlation between eleven growing Asian stock exchanges and developed markets. Similarly [40], argue that Asian markets were uniform and dominated by a strong market force and found no relationship between Asian markets and developed economies. Similarly [41], concluded the long and short-term relationship between the equities markets of 11 Asia-Pacific nations, including the Malaysian stock market and other important trading partners like Japan and the United States. Data was analyzed from July 1, 1996, to June 30, 1998, and found the short term and long term co-movement between them. [42] evaluated the interconnectedness of the stock markets of Australia, Hong-Kong, Japan, Korea, the U.K., and the U.S. based on the Co-integration tests and also of high intensity of the risk co-movement pattern between them at different time intervals.

[43] investigated the relationship of the stock markets of developed and emerging economies in the context of long-term relationships and found both short-term and long-term co-movement between these selected markets, such as India market has long-term co-movement with mature markets. A recent study by [44] looked at the correlation between the US and Argentina, Brazil, China, India, and Russia stock markets and found a strong cointegration between the selected markets due to the trade interdependence. [45] found the interrelationships between the markets of GCE countries. In that study, there was a period between June 2, 2005, and April 2, 2008, and high cointegration between the selected economies was found during the respective period. Moreover, they concluded that the cointegration between the stock markets varies due to the volume of the trade agreements, trade volume, and foreign direct investment.

[46] investigated the long-term relationship between the German and Central and Eastern European stock markets. This study also looked into the impact of various stock market characteristics, including size and volatility, as well as interest rate and inflation differentials, on integrating these markets into the global economy. [47] examined the South African stock market and found strong co-integration with the major global stock markets. Moreover, India, Singapore, and Malaysia’s equity markets are compared using stock prices from July 1997 to February 2005 to assess the long-term and short-term linkages. To see the co-integration [45], studied India and two other developed economies, Japan and the USA. They found a significant relationship between them due to the trade agreements. [48] conducted a study on the cointegration between Malaysia, Hong Kong, Taiwan, and South Korea. They found a solid linear cointegration between the stock markets of the selected economies due to the trade alliances prevailing in those days. On the ground of previous literature, we developed the following hypothesis,

***H1***. The Global Financial crisis significantly negatively impacted Malaysia’s stock market and trading partners pre- and post-crisis.

***H2***. The risk in the Malaysian stock market has significant positive co-movement with its trading partners pre- and post-crisis.

***H3*.** Malaysian stock market has significant positive causation with trading partner’s stock markets pre- and post-crisis.

## 3. Material and estimated methods

### 3.1 Data description and sample

We use the daily stock market indices data from 1^st^ January 1993 to 31^st^ December 2021 with 7565 observations for each country’s stock market. The stock market taken as a sample includes Malaysia, China, India, Indonesia, Pakistan, Singapore, the United States of America (USA), Germany, France, and the United Kingdom (UK). The selection of the stock markets is based on the trade flow and volume between these countries, like exports and imports. According to [49] that explained the price and the volatility linkage through the trade flow and trade volume. These selected countries are the most significant trading partners of Malaysia. The trade flow between Malaysia and the selected trading partners increased from 1993 to 2021. China is its biggest trading partner, with a trade volume of $423 Billion in 2019 and an export volume of $336 Billion. Malaysia’s second-largest trading partner is Singapore, with an export trade volume of $ 330 Billion and an Import trade volume of $261 Billion, which has been increasing since 1992.

Pakistan is also a trading partner of Malaysia, with an import trade volume of $2.5 Billion and an export of $ 1.1 Billion. It has an increasing trend in the trade volume. India has a trade volume of exports with Malaysia of $9.0 Billion and imports of $5.8 billion. The United Kingdom is a trading partner of Malaysia, with an import trade volume of $1.7 Billion and an export volume of $2.19 Billion. The United States is Malaysia’s third biggest trading partner, with a trade volume of imports of $165 Billion and a trade volume of exports of $231 Billion. Japan is Malaysia’s fourth most significant trading partner based on trade volume, with the primary export of all products with a volume of $157 Billion and imports of $153 Billion, an increasing trend compared to the previous years. Germany is a trading partner of Malaysia with a rising trend in trade volume, with the export of all products at $6.2 Billion and imports at $6.4 Billion. France is also a trading partner of Malaysia, with a trade volume of $1.5 Billion and import of $2.6 Billion with the increasing trend. Indonesia is also a trading partner of Malaysia, with a trade volume of exports of $7.4 Billion and imports of $9.3 Billion, with an increasing trend compared to the previous years.

Malaysia was selected as the base economy on the ground of different reasons. First, it has been a growing economy since 1986 but was affected in 1997–98. Secondly, Malaysia is selected on the grounds of regional proximity; Malaysia has not been influenced by other political factors such as war and border conflicts, etc. Data of indices (MSCI) is extracted for each stock market from the DataStream database using the University Utara, Malaysia Library access. The long-term time horizon is selected to investigate critical events in the world economy with more significant change. The selected period also includes the period of 1993 to 2021, which describes the increasing trend of oil prices globally, Mexican currency crisis (1994–95), Asian economic crisis (1997–98), Russian default (1998), major economic crisis (2007–09) and also the period of COVID 19. Nowadays, the period of COVID-19 is also a hot topic due to the lockdown of business activities globally, which has negative consequences on the global economy.

### 3.2 Estimated models

This study used different estimated models to obtain our study objectives. To attain our objectives, we used the complete wavelet approach. However, our applied approach is very suitable for three key reasons. First, this study covers OECD and emerging stock markets, which helps compare the emerging economy across other regions. Second, this is supported by the reasonably large sample size; other approaches are useless due to the large sample or manipulating the results on a large sample. However, our study approach is very suitable for large sampling sizes, especially in the time series. Third, by fulfilling the necessities of the research, the risk co-movement transfer from Malaysia to its trading partners.

#### 3.2.1 Time-varying volatility

As per the GARCH modeling, volatility clustering is one of the specific characteristics of the stock market return. Before the volatility analysis through GARCH Modeling, we should fulfill the GARCH assumption of the volatility clustering existing in the stock market return. Therefore, we use the GARCH (1,1) model to estimate the time-varying volatility for *r*_*t*_, a country’s stock market return:

$$r_{t}=\alpha +\beta r_{t-1}+\epsilon_{t}\;where,\;\epsilon_{t}|I_{t}∼N(0,\sigma_{t}^{2})$$ (1)

$$\sigma_{t}^{2}=\omega_{0}+\omega_{1}\epsilon_{t-1}^{2}+\omega_{2}\sigma_{t-1}^{2}.$$ (2)

Eq (1) indicates the average model equation, while Eq (2) indicates the conditional uncertainty that tracks transient fluctuations of the stock market, capturing the conditional volatility that encapsulates the time-variable uncertainties in the financial markets of our study. Our goal is to analyses both co-movement and volatility. To do this, we split our sample into the OECD and emerging economies to learn more about how risks are distributed across the two regions [50]. We investigate how Malaysia’s stock markets move in tandem with its trading partners in Asia and other regions. The lag selection is based on the VAR (vector autoregressive) model. We select the lag value that is 1, and that’s why our GARCH estimation is (1,1). According to [50], the lag selection should be based on SC and HQ when both parameters are significant at the same point, and less lag is suitable for an accurate result.

#### 3.2.2 Wavelet analysis

The wavelet method is a modern and advanced tool for analyzing time-series behavior in the time-frequency domain. The analysis of wavelet helps academics and practitioners to decompose a time-series (*ψu*, (*t*)) into several components that allow deducing information over time. In line with earlier works like [51, 52], a wavelet, *ψ*(⋅)∈*L*^2^(ℝ), a real-valued or a complex-valued function defined over the real axis is expressed in the following:

$$\psi (t)=\frac{1}{\sqrt{s}}\psi \left(\frac{t-u}{s}\right)$$ (3)

in which $1/\sqrt{s}$ represents the factor of normalization ensuring that ‖*ψ*_*u*,*s*_‖^2^ = 1, where you represent the position of the respective wavelet and s represents the parameter for scale dilation. The wavelet specified by Morlet is defined as:

$$\psi_{0}^{M}(t)=\pi^{-1/4}e^{i\omega_{0}t}e^{\frac{{-t}^{2}}{2}}$$ (4)

where *ω*_0_ represents the wavelet’s central frequency that must be chosen appropriately to satisfy a good balance between time and frequency localization [53, 54].

#### 3.2.3 Continuous wavelets

The continuous wavelet transform defined in [53, 54] (CWT), *W*_*x*_(*u*, *s*) through a *ψ*(.) projection on the time-series as:

$$W_{x}(u,s)=\int_{-\infty }^{\infty }x(t)\frac{1}{\sqrt{s}}\bar{\psi (\frac{t-u}{s})dt}$$ (5)

where *ψ*(.) denotes the specific wavelet. The CWT could combine the function *x*(*t*)∈*L*^2^(ℝ) such that

$$x(t)=\frac{1}{c_{\psi }}\int_{0}^{\infty }[\int_{-\infty }^{\infty }W_{x}(u,s)\psi_{u,s}(t)d_{u}]\frac{d_{s}}{S^{2}},s>0.$$ (6)

The variance for the power spectrum can be specified as follows:

$$x(t)=\frac{1}{c_{\psi }}\int_{0}^{\infty }[\int_{-\infty }^{\infty }|W_{x}{\left(u,s\right)}^{2}|d_{u}]\frac{d_{s}}{S^{2}}.$$ (7)

#### 3.2.4 Cross-wavelet transform, wavelet coherence, and phase differences

This paper employs the Cross-Wavelet Power (hereafter, XWP) to locate the high market price-co-movement regions in the time-frequency domain. The two-signal cross-wavelet can be defined through the spectrum of cross-wavelet ($W_{n}^{XY}(s)$) as:

$$W_{n}^{XY}(s)=W_{n}^{X}(s)W_{n}^{Y^{*}}(s),$$ (8)

where $W_{n}^{Y*}(s)$ represents the complex conjugate of $W_{n}^{X}(s)$. $W_{n}^{XY}(s)$. The theoretical distribution of the cross-wavelet power of two signals with power spectra $P_{\kappa }^{X}$ and $P_{\kappa }^{Y}$ is given in the following form:

$$D(\frac{\left|W_{n}^{X}(s)W_{n}^{Y^{*}}(s)\right|}{{\;}^{\sigma }X^{\sigma }Y}<p)=\frac{Z_{v}(p)}{v}\sqrt{P_{K}^{X}P_{K}^{Y}},$$ (9)

where ^*σ*^*X* and ^*σ*^*Y* denote the standard deviations of *x* and *y*, *Z*_*v*_(*p*) represents the confidence interval with p to be the probability density function following a *χ*^2^ Distribution. The wavelet coherence is computed as:

$$R^{2}(u,s)=\frac{{\left|S(s^{-1}W_{xy}(u,s))\right|}^{2}}{S(s^{-1}{\left|W_{x}(u,s)\right|}^{2}).S(s^{-1}{\left|W_{y}(u,s)\right|}^{2})},$$ (10)

In the above equation, the smoothing parameter is denoted by *S*. The coefficient of squared wavelet-coherence (CSWC) satisfies the inequality condition of 0≤*R*^2^(*u*, *s*)≤1. *R*^2^(*u*, *s*) approaching one (zero) implies a high (weak) correlation. Due to the above reasons, the wavelet-coherence approach is considered the most appropriate method to inspect a variable in time and frequency domains. In addition, the two time-series phase-difference variables, that is, *ϕ*_*x*,*y*_. It can be used to distinguish between the phase-relationship. The phase difference defined below determines the positions in the pseudo-cycle:

$$\phi_{x,y}={tan}^{-1}\left(\frac{T\{W_{n}^{xy}\}}{R\{W_{n}^{xy}\}}\right)\;with\;\phi_{x,y}\in [-\pi ,\pi ].$$ (11)

As shown in Table 1, Arrows are designed to describe the phase and lead-lag relationships. Right (Left) pointing arrows indicate that the two variables correlate positively (negatively). Besides, an arrow’s right and up or left and down direction indicates that x(t) leads to y(t). Similarly, the left and up or right and down arrow movement indicates y(t) leads x(t).

**Table 1:** Descriptive statistics.

**Panel D 1993–2021**											
Description	MALAYSIA	CHINA	FRANCE	GERMANY	INDIA	INDONESIA	JAPAN	PAKISTAN	SINGAPORE	UK	USA
Mean	0.011	-0.002	0.021	0.021	0.040	0.037	0.006	0.013	0.009	0.012	0.032
Median	0.000	0.000	0.027	0.055	0.000	0.000	0.000	0.000	0.000	0.014	0.036
Maximum	23.263	14.036	10.363	11.125	16.423	16.829	13.062	14.199	10.974	9.265	11.043
Minimum	-24.159	-14.457	-13.150	-13.341	-13.740	-19.145	-10.435	-15.733	-9.833	-11.503	-12.922
Std. Dev.	1.263	1.792	1.318	1.367	1.458	1.764	1.291	1.651	1.191	1.095	1.147
Skewness	0.766	0.014	-0.245	-0.264	-0.287	-0.129	-0.203	-0.430	-0.036	-0.342	-0.456
Kurtosis	59.940	9.200	9.438	9.187	11.182	14.370	9.231	10.152	10.385	11.220	14.910
Jarque-Bera	1022683	12116	13139	12153	21207	40767	12291	16355	17193	21445	44972
Probability	0.000	0.000	0.000	0.000	0.000	0.000	0.000	0.000	0.000	0.000	0.000
Sum	84.781	-18.284	155.987	159.689	301.383	281.454	46.827	96.150	68.118	90.403	242.493
Sum Sq. Dev.	12063	24290	13133	14125	16088	23530	12599	20622	10727	9066	9959
Observations	7565	7565	7565	7565	7565	7565	7565	7565	7565	7565	7565
**Panel C 1997–98**											
Description	MALAYSIA	CHINA	GERMANY	FRANCE	INDIA	INDONESIA	JAPAN	PAKISTAN	SINGAPORE	UK	USA
Mean	-0.356	-0.314	0.027	0.011	-0.092	-0.358	-0.118	-0.165	-0.197	0.011	0.035
Median	-0.575	-0.388	0.160	0.015	0.000	-0.207	-0.118	0.000	-0.124	0.046	0.078
Maximum	23.263	12.725	5.594	6.076	7.288	16.829	6.814	14.199	10.974	3.493	4.859
Minimum	-24.159	-14.457	-7.532	-4.991	-5.590	-19.145	-5.099	-15.733	-8.999	-3.610	-6.967
Std. Dev.	3.904	3.325	1.655	1.443	1.597	3.729	1.427	2.837	2.056	1.122	1.256
Skewness	0.888	0.117	-0.749	-0.304	0.137	-0.205	0.248	-0.647	0.577	-0.248	-0.824
Kurtosis	14.395	5.533	5.099	4.790	4.428	7.336	5.228	9.237	8.848	3.707	9.330
Jarque-Bera	1812.04	88.16	90.64	48.70	28.80	258.52	71.02	552.76	484.10	10.17	582.93
Probability	0.000	0.000	0.000	0.000	0.000	0.000	0.000	0.000	0.000	0.006	0.000
Sum	-116.322	-102.614	8.750	3.580	-30.131	-117.124	-38.679	-53.894	-64.553	3.621	11.283
Sum Sq. Dev.	4968	3603	893	678	831	4533	664	2624	1379	410	514
Observations	327	327	327	327	327	327	327	327	327	327	327
**Panel B 2008–09**											
Description	MALAYSIA	CHINA	FRANCE	GERMANY	INDIA	INDONESIA	JAPAN	PAKISTAN	SINGAPORE	UK	USA
Mean	-0.099	-0.097	-0.120	-0.110	-0.047	-0.037	-0.149	-0.149	-0.124	-0.090	-0.081
Median	-0.009	0.000	-0.083	0.000	0.000	0.016	-0.030	0.000	-0.086	-0.032	0.006
Maximum	4.326	12.853	8.501	5.733	7.073	8.973	5.006	9.330	6.099	8.489	5.227
Minimum	-10.242	-10.813	-6.888	-7.386	-9.494	-8.008	-5.992	-5.122	-6.492	-5.549	-9.160
Std. Dev.	1.288	2.757	1.569	1.365	2.207	2.155	1.712	1.888	1.618	1.561	1.491
Skewness	-1.406	0.188	0.252	-0.291	-0.228	-0.174	-0.212	0.062	0.145	0.308	-0.666
Kurtosis	14.862	5.233	6.597	6.937	4.554	5.196	3.756	5.458	4.609	6.078	7.630
Jarque-Bera	2024.880	69.856	179.736	215.799	35.749	67.335	10.225	82.544	36.411	134.267	316.282
Probability	0.000	0.000	0.000	0.000	0.000	0.000	0.006	0.000	0.000	0.000	0.000
Sum	-32.360	-31.714	-39.217	-35.922	-15.211	-11.951	-48.748	-48.709	-40.467	-29.302	-26.543
Sum Sq. Dev.	540.848	2477.562	802.829	607.244	1587.950	1513.658	955.360	1161.785	853.852	793.945	724.436
Observations	327	327	327	327	327	327	327	327	327	327	327
**Panel A 2020–21**											
Description	MALAYSIA	CHINA	FRANCE	GERMANY	INDIA	INDONESIA	JAPAN	PAKISTAN	SINGAPORE	UK	USA
Mean	-0.017	0.078	0.008	0.027	0.066	-0.046	0.044	-0.089	-0.010	-0.041	0.073
Median	0.000	0.100	0.052	0.056	0.194	0.000	0.000	0.000	0.000	0.023	0.166
Maximum	6.794	4.870	8.058	9.900	8.459	14.444	7.056	4.931	6.504	8.494	8.983
Minimum	-5.523	-6.172	-13.150	-13.341	-13.740	-8.430	-5.691	-7.791	-7.411	-11.503	-12.922
Std. Dev.	1.130	1.565	1.841	1.813	1.789	2.056	1.312	1.653	1.411	1.690	1.981
Skewness	-0.192	-0.480	-1.273	-1.248	-1.760	0.547	-0.067	-1.149	-0.375	-1.048	-0.988
Kurtosis	9.329	4.199	13.850	15.530	17.810	12.074	7.330	7.974	9.432	12.460	13.507
Jarque-Bera	546.069	32.030	1687.105	2217.145	3147.506	1134.785	254.877	407.743	569.652	1275.350	1552.489
Probability	0.000	0.000	0.000	0.000	0.000	0.000	0.000	0.000	0.000	0.000	0.000
Sum	-5.547	25.404	2.627	8.829	21.588	-14.998	14.225	-29.121	-3.258	-13.264	23.780
Sum Sq. Dev.	414.771	795.694	1102.100	1067.762	1039.628	1373.342	559.717	887.581	647.300	927.765	1275.483
Observations	326	326	326	326	326	326	326	326	326	326	326

#### 3.2.5 Wavelet-based granger causality

Even though economic theory is built on two-time scales, examining the different periods is crucial since they have different causal links. Time series commonly contain high- and low-frequency components. This study uses a non-parametric method to assess the Granger causality in spectral density matrices produced via wavelet modification. Wilson-Burg spectral factorization and non-linear variance decomposition are employed [55]. The spectral matrix elements obtained by a wavelet transformation of a time series are measured using $S_{ab}={[W}_{Xa}(t,f)W_{Xb}(t,f{)}^{*}]$ where a = 1, 2; b = 1.2. Here *W*_*Xa*_(*t*, *f*) represent the continuous mother wavelet transformation employing the mother wavelet function, Ψ(*η*), which is articulated as:

$$W(t,s)=|S{|}^{0.5}\int_{-\infty }^{\infty }x(\eta )\Psi^{*}(\frac{\eta -1}{s})d\eta$$ (12)

* specifies a complex conjugate. The data’s time-frequency representation is obtained by varying the scale parameter s and decoding over time t, yielding the wavelet function’s location. This study chose the Morlet wavelet, which is a plane wave modulated by a Gaussian envelope, $\Psi (\eta )=\pi^{-1/4}\exp\left(\mathrm{i\omega \eta}\right)\exp\left({-\eta }^{2}/2\right)$ With *ω*≥6 as the wavelet function. The Gaussian envelop, exp(−*η*^2^/2) commendably confines the wavelet in time, and *ω* controls the time/frequency determination. The terms frequency and scale are used interchangeably (*s*≈*f*). The time-frequency domain resolution is inversely related, as shown by the fact that a more significant value improves frequency resolution but reduces time resolution [56]. Among wavelet types, the Morlet wavelet provides the best data time-frequency distribution. The cycle analysis process commonly makes use of it. The Morlet wavelet is a type of wavelet analysis that benefits from the varying periods of non-stationary data. It can detect high-frequency or short-term changes [57]. To factorize the spectral density matrix S into a collection of unique lowest phase (thus, stable inverse) functions, use the Wilson-Burg matrix factorization theorem [58].

$$S=\psi \psi^{*}$$ (13)

where * denotes the matrix adjoint, and *ψ* denotes the minimum-phase spectral density matrix factor, with $\psi (exp(if))=\sum_{k=0}^{\infty }A_{x}exp\;exp(ikf)$. Here, *A*_*k*_ equals $(\frac{1}{2\pi })\int_{-\pi }^{\pi }\psi (\exp\left(if\right))\exp\left(-ikf\right)df,$ where *ψ*(0) = *A*_0_, which is a real upper triangular matrix with constructive diagonal components. After an assessment of Eqs (4) and (6), we write the error covariance matrix as:

$$\Sigma =A_{0}A_{0}^{T}$$ (14)

Likewise, by rewriting Eq (6) as $S=\psi A_{0}^{-1}\;A_{0}\;A_{0}^{T}\;A_{0}^{-T}\;\psi^{*}$ and comparing Eqs (4) and (7), the transfer function can be rewritten as:

$$H=\psi A_{0}^{-1}$$ (15)

Here, ψψ* = HΣH* * = *, and *T* denotes the matrix transposition. Spectral matrix factorization is a vital and novel step to non-parametrically obtain *H* and *Σ* from spectral analysis. The Wilson-Burg algorithm is a widely used factorization method that achieves superb numerical efficiency. It eliminates the effort from *O*(*N*^2^) to *O*(*N*^3^) operation when carrying out factorization. The Wilson-Burg algorithm is a commonly used spectral density matrix factorization algorithm. The convergence theorem of [56] ensures validity. The noise covariance matrix and the transfer function in Eqs (14) and (15) produced from Wilson-Burg factorization into the spectral Granger causality formula in Eqs (14) and (15) are used to estimate non-parametric wavelet Granger causality.

We use a wavelet approach to determine the synchronization between the selected stock markets. Wavelets are excellent at capturing the non-stationary behavior and time-varying trends present in the stock volatility data. In the frequency-time domain, the wavelet can be used to analyze risk co-movements in OECD and developing stock markets [59, 60]. The cross-wavelet transforms and wavelet coherence are discussed in this study as tools for analyzing the cointegration between two-time series. Additionally, this study demonstrates how the Granger causality test can confirm causal linkages and evaluate the mechanical model of physical links between related time series. Red noise backgrounds are used to evaluate the statistical significance through Monte Carlo simulation techniques. Furthermore, shocks that affect the interrelationships between time series can be timed more precisely with the help of wavelets.

## 4. Results and discussions

### 4.1 Summary statistics

The time series regular stock price and the return graphs describe the changing means and volatility for the sampling period 1993 to 2021 and display the volatility clustering, an assumption of the research modeling.

Fig 1 above shows that all indices show a simultaneous decline in the stock market in response to the financial crisis of 1997–98, 2001, 2008, 2012, 2015, and 2020. The decline in China’s stock market was also observed in July 2015 due to the Devaluation of the China Stock market and its impact on China’s trading partners. However, higher trends have been observed since 2015 in Indonesia, Malaysia, the USA, and India than in other countries like China, Singapore, and China. The UK, France, Germany, and Pakistan trend pattern shows that the 2015 China currency devaluation has affected the market but does not follow the same pattern. The disparity in the trend of each stock with other country markets shows the low correlation between them. We can see the return volatility of each stock market concerning return in the above figure. Every selected market had volatility clustering during the financial crisis. Still, Malaysian return volatility was low as compared to the other stock markets during the financial crisis of 2008–9, but Malaysian return volatility was high during the financial crisis of 1997–98, which means that the global financial crisis of 1997–98 has more effect on Malaysian economy as compared to the global financial crisis of 2008–9. Some preliminary GARCH and wavelet assumptions justify this methodology’s selection and make them suitable for the current study.

**Fig 1:** Return volatility pattern of all selected markets.

The selected stock market returns’ descriptive statistics in Panel D (1993–2021), the Malaysian stock market index has an average return that is positive 0.011207, with a maximum value of 23.26283 and minimum -24.1591, the second lowest in the selected markets group. The positive return of Malaysia indicates the positive performance of the Malaysian stock market in the selected timeframe. China has a negative mean value of -0.00242, with a maximum of 14.03612 and a minimum of -14.4569, the lowest value in the group. It means China’s stock market performance is low due to the average stock market return in the respective time, indicating the loss in the selected timeframe. France, Germany, Pakistan, Indonesia, UK, and the USA have positive average returns, meaning these markets perform well due to the market structure. The Indian Stock market has an average return of 0.039839, the highest average return in the group during the selected period in panel D, which means that Indian Stock has approximately 4% average return earned on their investment during that period.

In Panel C, the Malaysian stock market index has an average rerun of -0.35573, which means that the Malaysian market faced a loss due to the financial crisis of 1997–98, with a minimum return of -24.1591 and a maximum of 23.26283 due to the high volatility due to bad news of the crisis shock. From the given data, we can conclude that in the selected period of panel C, Malaysian stock market performance is negative due to the financial crisis of 1997–98. In Panel C, all the selected markets have negative average stock returns except Germany, France, the UK, and the USA; these markets are developed and a small decline in their average return due to the financial shock. The crisis impacted all markets, including OECD stock markets, due to the negative average return on a specific day. Malaysia and Indonesia Stock markets have the lowest average return in the group, which is -0.35573 and -0.35818, respectively, which means that the financial shock of 1997–98 hit these economies very critically.

In panel B, the period of 2008–9, every stock market has a negative average stock return due to the global financial crisis 2008 9. Malaysia has an average stock return of -0.09896, China has -0.09698, Indonesia has -0.03655, Pakistan has -0.14896, and others have negative. Japan has a -0.14908 average return, the lowest in the selected group. Indonesia has better than all selected economies but has negative performance with an average return of -0.03655 during the 2 08–9 global financial crisis. In panel A, Malaysia has an average return of -0.01701, Indonesia -0.04601, Pakistan -0.08933, Singapore -0.00999, United Kingdom -0.04069, and other markets China, Japan, USA, France and Germany have a positive average return. It means that the negative average return stock markets faced the problem of COVID-19 critically by the lockdown in their business, and that’s why their performance goes to the negative but those countries that average return in this period is positive, it means that their supply chain is effective despite the pandemic crisis. In panel A, the country stock market with the highest average return in the selected group is China, with 0.077928. Pakistan’s lowest average return country has a negative average return of -0.08933. Due to these factors, China faced the first entry of COVID-19, but the government of China made innovative measures to promote its economy through different measures and controls.

The volatility or the fluctuation from its means of the stock prices can be measured through the calculation of the standard deviation of the sample. If volatility from its means is greater, there is a high risk in the stock prices. When we look at Panel D, the highest and lowest value of the standard deviation in the selected markets is 1.792002 and 1.094799, representing China and the United Kingdom, respectively. In Panel C, the stock price with the highest and lowest standard deviation values is 3.903887 and 1.122109, representing Malaysia and the UK, respectively, in the period of financial crisis 1997–98. Malaysia faced huge volatility or fluctuation in the stock prices due to the financial crisis of 1997–98, but the lowest fluctuation is found in the stock prices of the United Kingdom. In Panel B, China has the highest value of a standard deviation of 2.756789, and Malaysia has the lowest value of 1.288039; it means that during the Global financial crisis of 2008–9, China’s stock price fluctuated more as compared to the other economies in the group. Still, Malaysia has the lowest fluctuation, even with a negative average return of -0.09896. The highest and lowest standard deviation is being observed in Indonesia and Malaysia, representing 2.055643 and 1.129698, respectively, meaning that Indonesian Stock prices have greater return volatility than the selected markets. Malaysia has the lowest volatility due to the strong measures by the central government. All the selected markets, except the lowest and highest, go to approximately 1.5 value of standard deviation in their stock return.

The Skewness describes the normal distribution of data. If the skewness value is zero, then we can say that the data set is normally distributed. Before the run of the analysis, some assumptions of the model run should be fulfilled by the researchers. The data normal distribution is also necessary for the data analysis to minimize errors. A skewness may be a positive or negative value; if it is a positive skewness, it is suitable for the normal distribution of data because Skewness is the indicator of the normal distribution of the dataset. The negative skewness means the values are not suitable. In panel D, all the countries’ stock return skewness value except Malaysia and China is negative, which indicates the data set is unsuitable for normal distribution and frequently changes due to crisis. Similarly, Malaysia and China’s skewness value is positive, indicating a suitable normal distribution markets dataset.

In panel C, some countries, like Malaysia, China, India, Indonesia, Japan, and Singapore, have positive Skewness, indicating the suitable normal distribution of the dataset during the period of the financial crisis of 1997–98. On the other side, in the selected group, Germany, France, UK, USA, and Pakistan skewness value is negative, indicating a suitable value. Similarly, In panel B, Malaysia, Germany, India, Indonesia, and the USA had negative skewness in 2008–9, while other selected countries had positive skewness that indicated suitability. Same as in Panel A, all the country’s stock return skewness value is negative, indicating the non-suitable normal distribution of the financial market’s dataset in the period of COVID-19 due to the lockdown of the business activities, and the dataset shows the abnormal changes from the previous one due to pandemic.

The Kurtosis value in the descriptive statistics measures the probability in the tail of the bell shape of the normal distribution diagram. The kurtosis value should equal 3, which is helpful compared to the normal distribution. Our analysis considers that the Kurtosis value should be greater than 3, meaning the selected dataset is normally distributed.

The goodness of fit of the sample normally distributed data based on the Skewness and Kurtosis value is represented by the Jarque-Bera test. The Jarque-Bera test should be far from zero value. Jarque-Bera is also used to diagnose the normal distribution in datasets for large sample sizes. The significant value at a 1% level of significant is adjusted to reject the null hypothesis in our Jarque-Bera test analysis, and compared with the Kurtosis value, its Kurtosis value is less than three, then we indicate that the data is not normally distributed. There is a necessary assumption of the Generalized Autoregressive Conditional Heteroscedasticity (GARCH) Modelling.

Table 2 summarizes the correlation matrix of the sample. If a positive correlation existed between the two stock markets, then we can say that a common co-movement direction existed. In our sample countries, stock market correlation ranges from 0.0056 to 0.8523, respectively. Stock returns are below the value of 0.80, indicating weak co-movement and a lack of multi-collinearity. In our correlation matrix, the correlation value between France and the UK is above 0.80, indicating the strong co-movement between these countries’ stock markets return in panel D; both countries belong to the OECD economies. Same as in the period of crisis of 1997–98, the correlation value between Germany-France and France-UK is above 0.80, indicating strong cointegration. However, Malaysia- Singapore has greater value in the emerging economies but less than 0.80.

**Table 2:** Correlation matrix.

**Correlation Panel D 1993–2021**											
Countries	MALAYSIA	CHINA	FRANCE	GERMANY	INDIA	INDONESIA	JAPAN	PAKISTAN	SINGAPORE	UK	USA
MALAYSIA	1.000										
CHINA	0.334	1.000									
FRANCE	0.160	0.285	1.000								
GERMANY	0.158	0.286	0.856	1.000							
INDIA	0.187	0.336	0.286	0.264	1.000						
INDONESIA	0.311	0.370	0.204	0.197	0.282	1.000					
JAPAN	0.251	0.406	0.284	0.262	0.247	0.278	1.000				
PAKISTAN	0.095	0.076	0.053	0.051	0.116	0.080	0.068	1.000			
SINGAPORE	0.422	0.539	0.371	0.360	0.377	0.426	0.430	0.104	1.000		
UK	0.185	0.297	0.850	0.777	0.283	0.206	0.285	0.048	0.380	1.000	
USA	0.041	0.174	0.536	0.549	0.180	0.089	0.130	0.018	0.214	0.518	1.000
**Panel C 1997–98**											
Countries	MALAYSIA	CHINA	GERMANY	FRANCE	INDIA	INDONESIA	JAPAN	PAKISTAN	SINGAPORE	UK	USA
MALAYSIA	1.000										
CHINA	0.377	1.000									
GERMANY	0.177	0.258	1.000								
FRANCE	0.175	0.177	0.752	1.000							
INDIA	0.172	0.233	0.199	0.206	1.000						
INDONESIA	0.324	0.327	0.234	0.201	0.209	1.000					
JAPAN	0.253	0.299	0.350	0.394	0.109	0.292	1.000				
PAKISTAN	0.159	0.170	0.130	0.126	0.049	0.080	0.121	1.000			
SINGAPORE	0.467	0.522	0.303	0.280	0.206	0.417	0.322	0.303	1.000		
UK	0.272	0.247	0.704	0.764	0.221	0.203	0.377	0.126	0.322	1.000	
USA	-0.062	0.014	0.401	0.463	0.113	-0.035	0.110	0.011	0.075	0.455	1.000
**Panel B 2008–09**											
Countries	MALAYSIA	CHINA	FRANCE	GERMANY	INDIA	INDONESIA	JAPAN	PAKISTAN	SINGAPORE	UK	USA
MALAYSIA	1.00										
CHINA	0.52	1.00									
FRANCE	0.31	0.34	1.00								
GERMANY	0.31	0.33	0.95	1.00							
INDIA	0.40	0.62	0.40	0.40	1.00						
INDONESIA	0.52	0.62	0.28	0.29	0.49	1.00					
JAPAN	0.48	0.65	0.34	0.33	0.47	0.43	1.00				
PAKISTAN	0.14	0.04	0.07	0.05	0.14	0.08	0.12	1.00			
SINGAPORE	0.54	0.75	0.51	0.47	0.62	0.62	0.62	0.09	1.00		
UK	0.31	0.37	0.94	0.90	0.41	0.30	0.33	0.05	0.52	1.00	
USA	0.02	0.09	0.54	0.50	0.14	0.15	0.05	0.04	0.18	0.52	1.00
**Panel A 2020–21**											
Countries	MALAYSIA	CHINA	FRANCE	GERMANY	INDIA	INDONESIA	JAPAN	PAKISTAN	SINGAPORE	UK	USA
MALAYSIA	1.00										
CHINA	0.44	1.00									
FRANCE	0.37	0.49	1.00								
GERMANY	0.36	0.50	0.95	1.00							
INDIA	0.51	0.52	0.59	0.55	1.00						
INDONESIA	0.44	0.35	0.34	0.30	0.51	1.00					
JAPAN	0.38	0.42	0.46	0.45	0.34	0.29	1.00				
PAKISTAN	0.30	0.22	0.25	0.26	0.39	0.36	0.10	1.00			
SINGAPORE	0.59	0.53	0.56	0.55	0.67	0.47	0.57	0.25	1.00		
UK	0.29	0.47	0.91	0.88	0.54	0.28	0.46	0.19	0.53	1.00	
USA	0.16	0.49	0.66	0.67	0.39	0.31	0.31	0.18	0.36	0.66	1.00

On the other hand, some stock markets show less value of the correlation between them that seems more robust across developing countries, while smaller between OECD and emerging economies. Hence, we can consider these points in the diversification opportunity across the regions. By keeping these points in mind, we can diversify our portfolio and earn the maximum expected return on the given investment by minimizing the risk.

### 4.2 Wavelet transformation estimates and discussion

#### 4.2.1 Cross wavelet transformation of emerging and OECD countries

When localized similarities are present, the typical feature extraction uses the Cross Wavelet Transform (XWT) approach. This method requires fewer parameters than the other methods for classifying timeframe features into normal and abnormal classifications. Additionally, this method can produce more precise results because it is compatible with loud surroundings. Due to its capacity to manage the imaginary portion of the input without employing the absolute function, it also keeps the information on the phase. Figs 2–5 represent the XWT across the countries’ stock market indices return.

**Fig 2:** Cross-wavelet power spectra of selected stock markets (Panel D 1993–2021): Cross- wavelet power spectra are considered significant at 5% under the red noise prediction defined by Monte Carlo. The two variables have a positive relationship if the arrows are toward the right. Suppose the arrow is towards the right and up. In that case, the first variable leads, and there is a positive relationship, or if arrows are toward right and downward, the variables first are lagging and positive. On the other side, if the arrows are toward left and up, the first variable is lagging, and the relationship between variables is negative, or if the arrows are toward left and down, then the variable is leading, and the correlation is negative.

**Fig 3:** Cross-wavelet power spectra of selected stock markets during crisis 1997–98 (Panel C): Cross-wavelet power spectra are considered significant at 5% under the red noise prediction defined by Monte Carlo. Two variables have a positive relationship if the arrows are toward the right. Suppose the arrow is towards the right and up. In that case, the first variable leads, and there is a positive relationship, or if the arrows are towards right and downward, the variables first are lagging and positive. On the other side, if the arrows are toward left and up, the first variable is lagging, and the relationship between variables is negative, or if the arrows are toward left and down, then the variable is leading, and the correlation is negative.

**Fig 4:** Cross-wavelet power spectra of selected stock markets during crisis 2008–09 (Panel B): Cross-wavelet power spectra are considered significant at 5% under the red noise prediction defined by Monte Carlo. The two variables have a positive relationship if the arrows are toward the right. Suppose the arrow is towards the right and up. In that case, the first variable leads, and there is a positive relationship, or if arrows are toward right and downward, the variables first are lagging and positive. On the other side, if the arrows are toward left and up, the first variable is lagging, and the relationship between variables is negative, or if the arrows are toward left and down, then the variable is leading, and the correlation is negative.

**Fig 5:** Cross-wavelet power spectra of selected stock markets during the pandemic COVID-19 2020–21 (Panel A): Cross- wavelet power spectra are considered significant at 5% under the red noise prediction Monte Carlo defines. If the arrows are toward the right, two variables have a positive relationship. Suppose an arrow is towards the right and up. In that case, the first variable *is* leading, and there is a positive relationship, or if the arrows are towards right and downward, the variable first is lagging and has a positive relationship. On the other side, the first variable is lagging if the arrows are toward the left and up. The relationship between variables is negative, or if the arrows are towards the left and down, the variable leads, and the correlation is negative.

Moreover, we make four panels based on the crisis, considering D, C, B, and A, respectively. Panel D represents the period from 1993 to 2021. Panel C represents the time domain of the crisis period of 1997–98, the period of the Asian financial crisis. Moreover, panel B represents the period of 2008–09, the Global financial crisis. Panel A represents the time domain of the COVID-19 2020–2021 respectively. It should be emphasized that the arrows represent phase information that enables us to comprehend how various global markets interact with Malaysian markets.

The in-phase relationship in all selected country pairs is shown in Fig 2, related to Panel D (1993–2021), indicated by the arrows towards the right, which can be found in the numerous significant regions. In panel D, the pair Malaysia- India is an in-phase relationship during the period of the crisis 2008–09, with Malaysia as the leading effect at the low-frequency domain (32–128), but during the COVID-19 pandemic, both markets are in-phase relationship, and Malaysia is lagging, and India is leading on the Malaysia stock market, It means that during the financial crisis 2008–9, the Malaysian stock market drives Indian market but this seen is opposite in COVID-19 period.

In the pair of Malaysia-China, a high level of covariance is found between two stock market risks in the period of 1993 to 1999 at both high and low frequency domain, indicating the in-phase relationship between these two-stock market risks and Malaysia is leading effect, arrows are right and upward. The same level of covariance was observed in 2008–9 and 2020–21, and Malaysia is leading the China stock market risk at different frequency domains.

Similarly, a different pattern of market risk behavior is being observed in the two pairs of Malaysia-France and Malaysia-Germany, where both market risks are in phase, and Malaysia is lagging from 1993 to 2012 at the high frequency of (1024–2048), indicating the high level of the covariance between the risk of these selected countries and Malaysia is lagging because arrows are right and downwards. In 2008–9 and 2020–21, there is also covariance between these stock markets’ risk at low frequency, with Malaysia’s leading effect during 2020–21.

In addition, quite a similar pattern is found for the Malaysia-US pair; the significant in-phase relationship is shown during 2020–21 only, and Malaysia is the leading effect in that period. However, the same pattern of risk is found in the pairs of Malaysia-Japan and Malaysia-Singapore, indicating the in-phase relationship between risks and Malaysia is leading (lagging) from 1993 to 1994, 1995 to 2016, and 2020–21. High levels of covariance are also shown in these pairs during the financial crisis period of 1997–98 and 2008–9.

In the pair of Malaysia-Indonesia, we found the covariance during 2008–9 and 2020–21 at a medium level of the frequency domain, indicating the in-phase relationship with Malaysia is the leading effect. The arrows are right(upward). In the pair of Malaysia- Pakistan, in-phase relations are shown between these two stock market risks, indicating the high level of covariance between these two stock market risks; Malaysia is leading to the risk of Pakistan stock market from 1997 to 2008, 2008–9 and 2020–21 at the high, medium and low-frequency domain, means the high, medium, low level of covariance between the risk are found between the pairs.

Similarly, the same Parten is found between the Malaysia-USA stock market risk pair, where in-phase relationships are found. Still, Malaysia has a lagging effect from 1993 to 1997, 1997–98, and 2008–9 at low, medium, and high-frequency domains. This finding shows that the positive relationship between the time series USA stock market drives Malaysia. From our findings of Panel D, we show that Malaysia’s stock market risk is correlated with all trading partners during the crisis period and also after the crisis period, where Malaysia’s stock market risk drives the other trading partners stock market risk and sometimes other trading partners stock market risk drives the Malaysian stock market risk at different frequency levels and at different time domains.

Additionally, high levels of covariance are shown in XWT transformation for all emerging and OECD stock market pairs with Malaysia from 1993 to 2021; we denoted it as panel D in Fig 2. Our findings are consistent with the findings of [61–63]. We also found the co-movement in risk of some degree between Malaysia and its trading partners at low, medium, and long horizons in panel D.

In panel C (1997–98), the covariance between Malaysia-India, Malaysia-USA, Malaysia-France, Malaysia-Germany, Malaysia-Japan, and Malaysia-Pakistan- Malaysia-UK is seen positive from July to September 1997 in high frequency. We make the three months for finding the relationship between them according to the quarterly effect. In these pairs, Malaysia is leading effect, which means that in the crisis period from July to September 1997, the stock markets of India, USA, France, Germany, Japan, Pakistan, and the UK are driven by Malaysia due to leading effect, indicating arrows are right (upwards). In the pair Malaysia-China, there is also positive covariance from July to September 1997, but Malaysia has a lagging effect due to the arrows being right (downwards). An in-phase (positive) relationship is found only in Malaysia-Singapore and Malaysia-Indonesia. During December 1997, all the pairs were in a phase relationship, showing the positive covariance between them. During September 1998, all the selected pairs were in an in-phase (positive) relationship. From September to October 1998, Malaysia-Singapore Malaysia-India pairs, in which Malaysia is lagging effect at a higher frequency due to the trade fluctuation between them. Our results consisted of the findings of [64], also opposite to those of [65], which shows the negative covariance between selected markets in that period. In panel A (for the period 2020–21), in all the selected pairs, risk covariance is positive between them from March to August 2020, indicating that in the period of the COVID-19 disease, one economy transferred the financial risk to another economy. All the pairs show a high level of covariance from March to August 2020, and that’s why co-movement between the stock market is high in that period.

#### 4.2.2 Wavelet coherence transformation of emerging and OECD countries

Figs 6–9 exhibit wavelet coherence results at different intervals. It is shown that overall, the Malaysia stock market risk moves significantly with its emerging and OECD trading partners. In addition, a relatively large portion of the wavelet coherence area often turns into the region of core of influence (COI), which represents the significant, with left to right turns arrows, which indicates that Malaysia is in-phase (Positive covariance) with its all-selected trading partners.

**Fig 6:** Wavelet coherence of selected stock markets during crisis 1993–2021 (Panel D).

**Fig 7:** Wavelet coherence of selected stock markets during Crisis 1997–98 (Panel C).

**Fig 8:** Wavelet coherence of selected stock markets during crisis 2008–09 (Panel B). Wavelet Coherence is considered significant at 5% under the red noise prediction defined by Monte Carlo. The two variables have a positive relationship if the arrows are towards the right. Suppose the arrow is towards the right and up. In that case, the first variable leads, and there is a positive relationship, or if arrows are toward right and downward, the variables first are lagging and positive. On the other side, if the arrows are toward left and up, then the first variable is lagging, and the relationship between variables is negative, or if the arrows are toward left and down, then the variable is leading, and the correlation is negative yet.

**Fig 9:** Wavelet coherence of selected stock markets during crisis 2020-2021(Panel A) in panel C (1997–98), there is a high level of co-movement being found between the pairs Malaysia-China and Malaysia-Singapore; co-movement is high from October 1997 to October 1998 at medium and high-frequency domain because arrows are right at both frequency domains. In pairs, Malaysia-Pakistan, Malaysia-UK, Malaysia-Japan, Malaysia-France, and Malaysia-Indonesia in-phase relationships are being observed from June 1997 to August 1997 at frequency domain, indicating the short-run relationship between the risk of these stock market in the period of financial crisis and findings are similar with [51, 68]. The Malaysia-India Pair has high co-movement, and an in-phase relationship is observed from October 1998 to December 1998.

In Panel D (1992–2021), as the emerging trading partners for the couple Malaysia-China, Malaysia-Pakistan, and Malaysia-Indonesia, the right arrows indicate the positive covariance between them at a higher frequency domain from 1993 to 2021; in this way, our findings are consistent with the result of [66] that China, Malaysia, and Indonesia stock market risk are correlated at high frequency due to the trade agreements between them.

The covariance between emerging and OECD economies is very interesting for both regions. The risk covariance pattern between the pair Malaysia-Germany, Malaysia-UK, and Malaysia-France is positive, indicating the arrows are right (downwards) from 1993 to 2021, showing that Malaysia is lagging the Stock market of Germany, France, and the UK at a higher frequency. Still, during 2020–21, they had a high-risk covariance level.

In addition, in the pair of Malaysia-US, there is an in-phase relationship being seen in the period of 1997–98, 2007, and 2020 for the short run at a low frequency that shows the low level of the covariance due to the US and China Trade conflicts, China is the trade agreement with Malaysia already. In this context, our findings are consistent with the findings of [67]) that Malaysia and China are cointegrated with the USA at low frequency due to the conflicts. High co-movement was found between Malaysia and Japan at both medium and high-frequency domains from 1993 to 2021. In the pair of Malaysia-Singapore, positive cointegration is found between the risk of the stock markets at a low, medium, and high-frequency domain, indicating that the arrows are right due to the large trading volume between them. The in-phase relationship between the couple Malaysia-India during 2008–9 and 2020–21 at medium frequency domain considers the weak relationship in the selected group.

In panel A (2020–21), all the selected couples have an in-phase(positive) significant relationship, indicating the arrows are right and up(down), showing the leading and lagging risk of the Malaysia stock market for the time January 2020 to June 2021. Malaysia has to lead in the couple Malaysia-France and Malaysia-Japan during March 2020 because the arrows are right and up. Still, Malaysia lags in Malaysia-Indonesia and Malaysia-China pairs because the arrows are from October to December 2021.

### 4.3 Robustness: Wavelet-based Granger causality test

To complement our findings of the XWT and WCOH using the robustness test, we applied a wavelet-based Granger causality test using the four frequency domains (D1, D2, D3, and D4), and the results are exhibited in Table 3. Fig 10 also shows the directions of the causality between the selected stock markets. In our findings, most of the selected market has bi-directional causalities between Malaysia’s stock market and its trading partners. Still, the frequency domain varies from one pair to another pair or from one region to another. In particular, we find the bi-directional causation between the Malaysia stock market and the US, UK, France, Germany, Indonesia, and Singapore in the D1 frequency domain, corresponding to the short and long horizons. In addition, we find the unidirectional causality transfer from India and Pakistan, where both countries’ stock markets caused the Malaysia stock market due to the trading that existed between them. These findings confirm the strong correlation between them over the D1 frequency domain.

**Fig 10:** Wavelet Granger causality Malaysia vs. Selected markets.

**Table 3:** Granger causality test for emerging and OECD economy at various frequencies.

**Frequency Domain**	**Independent Variable**	**Dependent Variable**										
**D1**	***COUNTRY***	***MALAYSIA***	***FRANCE***	***GERMANY***	***INDIA***	***INDONESIA***	***JAPAN***	***CHINA***	***PAKISTAN***	***SINGAPORE***	***UK***	***USA***
	MALAYSIA		28.6557***	26.7694***	3.80154	3.02885**	0.60684	1.71034	0.0698	2.88212*	33.8582***	38.4182***
	FRANCE	75.9992***		0.0682	4.51507**	67.8841***	424.532***	120.442***	10.5533***	85.3534***	2.29458	53.4729***
	GERMANY	70.0670***	17.3533***		12.5668***	50.521***	387.968***	115.541***	7.52839***	101.457***	4.06290**	32.0487***
	INDIA	14.1105***	4.86897***	6.15997***		11.7796***	28.273***	3.041**	2.29766	0.13490	6.26184***	23.5285***
	INDONESIA	9.65302***	17.1649***	11.8088***	2.03964**		1.3804	2.867*	0.00179	6.95935***	23.9739***	37.4060***
	JAPAN	0.43267	104.655***	112.361***	13.8025***	2.28665		4.88667***	1.40205	14.0055***	98.4597***	187.247***
	CHINA	0.89978	41.6071***	49.412***	10.122***	5.143***	10.9336***		0.32728	18.5211***	28.4779***	80.8209***
	PAKISTAN	3.10963**	10.1536***	4.55114**	0.64473	5.18940***	1.27871	0.15352		1.29909	8.35943***	9.00903***
	SINGAPORE	11.5834***	23.7754***	29.0600***	2.19485	1.95247	32.7822***	11.8897***	1.11372		28.5613***	87.1038***
	UK	85.2226***	8.89413***	2.40883*	7.52932***	68.0097***	442.307***	114.61***	11.6413***	105.112***		65.3502***
	USA	134.802***	213.191***	141.525***	39.4526***	126.872***	525.209***	214.422***	9.66359***	260.381***	215.185***	
**D2**	***COUNTRY***	***MALAYSIA***	***FRANCE***	***GERMANY***	***INDIA***	***INDONESIA***	***JAPAN***	***CHINA***	***PAKISTAN***	***SINGAPORE***	***UK***	***USA***
	MALAYSIA		5.71866***	6.51985***	0.29738	3.06033**	2.16027	14.7231***	0.06581	0.95483	6.71971***	2.62718*
	FRANCE	21.3409***		23.6925***	24.5467***	36.1723***	206.325***	83.1279***	0.48017	48.388***	0.37406	14.8087***
	GERMANY	18.6352***	21.8052***		13.9922***	18.8025***	211.828***	80.4971***	0.47477	36.5117***	9.07076***	4.71015***
	INDIA	1.34287	2.68403*	1.35587		3.11801**	25.4501***	9.60525***	0.94194	0.09472	3.8866**	0.40824
	INDONESIA	19.7424***	6.71043***	4.74873***	0.89180		4.23277**	13.2238***	0.34392	6.18031***	4.79488***	2.54911*
	JAPAN	3.18695**	17.5963***	14.4197***	6.71078***	2.11674		1.70311	1.10235	3.44271**	19.9438***	11.2431***
	CHINA	21.5171***	5.86958***	11.1162***	9.6574***	2.20801	5.42748***		1.13144	16.1407***	2.91681*	8.28519***
	PAKISTAN	0.10424	9.97116***	5.13841***	0.55164	0.20960	1.40741	0.49115		0.55134	6.67498***	6.68089***
	SINGAPORE	4.31391**	0.83394	4.08216**	3.18682**	5.75960***	36.4177***	24.6301***	1.12653		2.12085	5.10276***
	UK	18.2857***	4.59388**	6.93552***	19.4852***	31.1229***	166.298***	57.0599***	0.73125	41.5295***		17.8413***
	USA	67.3852***	158.816***	115.914***	49.1388***	82.9117***	390.367***	165.877***	3.35795**	163.698***	172.341***	
**Frequency Domain**	**Independent Variable**	**Dependent Variable**										
**D3**	***COUNTRY***	***MALAYSIA***	***FRANCE***	***GERMANY***	***INDIA***	***INDONESIA***	***JAPAN***	***CHINA***	***PAKISTAN***	***SINGAPORE***	***UK***	***USA***
	MALAYSIA		0.67136	0.27848	3.76825**	5.46947***	2.74132*	4.5931**	11.7335***	3.6397**	0.17766	0.79647
	FRANCE	36.3167***		8.93080***	19.5716***	12.1629***	159.689***	20.4713***	1.82804	21.9447***	11.2791***	8.3524***
	GERMANY	31.6780***	1.77589		21.5294***	17.5858***	144.273***	11.3062***	1.06242	27.2522***	10.3773***	6.05603***
	INDIA	9.41455***	1.10099	0.30308		5.21466***	8.79452***	2.94943*	1.7399	0.62155	1.00675	0.49012
	INDONESIA	14.7413***	7.60283***	8.34136***	0.52667		8.34424***	0.99076	4.23202**	0.2548	2.01955	5.26463***
	JAPAN	8.07308***	0.34113	0.26327	2.25932	6.04226***		5.69743***	3.26832**	4.94862***	4.2398**	3.12301**
	CHINA	40.9882***	2.66644*	4.34339**	0.28341	1.64833	9.22877***		8.37448***	1.69116	1.09767	2.29522
	PAKISTAN	12.9557***	2.25964	3.05106**	9.50798***	5.80874***	2.17087	4.27675**		2.35309*	2.92891*	0.18028
	SINGAPORE	20.8068***	3.15608**	2.99052*	2.56655*	4.64778***	30.6046***	4.08046**	10.197***		3.42441**	2.55878*
	UK	32.8545***	11.8029***	14.1045***	20.4557***	18.1974***	154.407***	37.7490***	1.3173	21.3149***		1.10527
	USA	88.3633***	166.451***	127.675***	50.6238***	42.4667***	283.792***	105.794***	3.74623**	133.248***	151.93***	
**D4**	***COUNTRY***	***MALAYSIA***	***FRANCE***	***GERMANY***	***INDIA***	***INDONESIA***	***JAPAN***	***CHINA***	***PAKISTAN***	***SINGAPORE***	***UK***	***USA***
	MALAYSIA		1.18269	0.90002	1.22322	1.12337	2.22936	7.74383***	2.85105*	0.46287	4.02973**	0.2769
	FRANCE	21.1854***		1.7694	4.15802**	17.6496***	121.185***	25.4856***	17.1764***	42.8507***	2.25643	3.48096**
	GERMANY	28.5271***	0.88988		14.4717***	24.8448***	123.165***	40.1521***	15.9035***	57.2591***	3.63715**	9.13691***
	INDIA	3.25677**	3.47653**	1.16248		5.16604***	17.4677***	3.58501**	10.0019***	1.72061	2.15458	0.56198**
	INDONESIA	17.0644***	1.82212	4.07687**	0.68922		7.51116***	0.44116	7.08634***	1.90852	2.26426	2.4693*
	JAPAN	0.85549	7.40225***	13.3034***	4.67244***	3.87664**		6.50018***	4.13203**	2.93250*	14.0712***	1.17098
	CHINA	0.0537	1.00142	3.12835**	0.73845	1.00117	8.60384***		10.9483***	0.44276	2.2436	2.19754
	PAKISTAN	4.18613**	1.15942	0.31093	0.62048	0.71407	2.64772*	0.57068		1.36098	2.33079*	1.15827
	SINGAPORE	5.17499***	0.32545	0.37698	1.83741	10.8303***	13.7522***	0.76095	9.14092***		1.37432	0.7737
	UK	16.4921***	3.16723**	1.45144	8.91715***	14.5824***	101.330***	17.9989***	17.5267***	47.8071***		5.87309***
	USA	39.7472***	65.6574***	45.9539***	22.5265***	28.327***	169.606***	44.6668***	24.8038***	89.6227***	74.6483***	
***Frequency Domain***	***Independent Variable***	***Dependent Variable***										
**Original**	***COUNTRY***	***MALAYSIA***	***FRANCE***	***GERMANY***	***INDIA***	***INDONESIA***	***JAPAN***	***CHINA***	***PAKISTAN***	***SINGAPORE***	***UK***	***USA***
	MALAYSIA	-	4.7307	3.0653	9.8700	50.6917***	5.6539	18.311***	8.1884	19.5525***	6.7328	2.1507
	FRANCE	21.6337***	-	22.081***	26.1415***	18.4011*	24.9588***	14.0096**	8.2880	13.3823*	37.4406***	12.0193*
	GERMANY	17.7834***	13.5710**	-	30.4171***	33.1515***	10.2059	15.3847***	2.4271	12.4512*	10.5856	11.6200
	INDIA	17.9042***	6.1672	7.9953	-	12.3027*	7.2776	11.9493*	22.7252***	11.8569*	14.5220**	12.7171*
	INDONESIA	69.8378***	19.3386***	12.7047*	4.4243	-	6.2905	19.1970***	8.2145	9.5827	10.6620	12.2390*
	JAPAN	20.7662***	3.1915	12.2572*	21.0298	47.3353***	-	71.4622***	4.4740	54.2252***	15.6457**	6.71831
	CHINA	36.5633***	9.387	14.6043**	13.0117*	17.5991*	16.112**	-	9.9395	24.2604***	3.7647	4.6794
	PAKISTAN	18.6574***	17.0594***	5.7103	6.5377	20.8076***	3.1609	4.9337	-	5.7345	14.9156**	11.8055*
	SINGAPORE	12.5824*	7.4685	9.7981	10.2697	20.8210***	15.5846**	7.5710	7.1126	-	5.0112	8.7894
	UK	23.4694***	26.7443***	23.3432***	13.5713*	9.4483	32.7390***	35.5893***	11.2170	34.9255***	-	15.6891**
	USA	248.4180***	659.2065***	530.6530***	178.9931***	262.8604***	601.3178***	402.7803***	21.6220***	571.5506***	787.252***	-

Note. level of significance is 1%, 5%, and 10%, respectively and represented by ***, ** and *

Similarly, we find bi-directional causality in D2 and D3 between the Malaysia-Indonesia and Malaysia-China. In a similar pattern, there is unidirectional causality between Malaysia, Japan, and Singapore, and there is also bi-directional causality between Malaysia and the USA, France, Germany, and China in the D1 frequency domain. In addition, in the D3 frequency domain, bi-directional causality between Malaysia and Japan, India, Pakistan, China, and Singapore found, also unidirectional causality find between Malaysia and UK, USA, France, Germany, where these countries stock market causes the Malaysia stock market over the D3 frequency domain. Interestingly, causality results show evidence of only two pairs of bi-directional causality found between Malaysia-Pakistan and Malaysia-UK in frequency domain D4. All the other countries except Japan cause Malaysia to be in the D4 frequency domain. In the original frequency domain from 1993 to 2021, bi-directional causality was found between Malaysia-Singapore, Malaysia-Indonesia, and Malaysia and China couples; the rest of the countries had unidirectional causality with Malaysia and caused to Malaysia stock market at the overall selected time domain.

The Granger causality test shows evidence of significant bi-directional and unidirectional causalities transfer from Malaysia to other trading partners and vice versa over all the selected frequency domains. This is consistent with the idea that there will not be an issue of the leader position between the Malaysian stock market and its trading partners in the long run, except for Indonesia, Singapore, and China. Similarly, when we compare the OECD country’s causality, we find the unidirectional causality transfer from the OECD economy to Malaysia on the different time horizons.

These findings imply that the temporary shocks of the developed or OECD country’s stock markets directly impact the Malaysian stock market, extending to the longer scale. At the same time, proximity does not affect stock market correlation as Malaysia and its trading partners need longer to absorb each stock market shock and adjust their prices accordingly. To sum up, our time-frequency domains causality analysis (D1, D2, D3, and D4) sheds light on the time the Malaysian market requires to interact with its trading partners and the nature of the lead-lag relationship. This time-frequency is very helpful for investors to decide on the investment in Malaysian stock market by considering the shock effect and its captured period.

### 4.4 Robustness: Dynamic conditional correlation GARCH

When one univariate time series has impact on the other univariate time series then we can say that multivariate analysis existed. Same as, when one stock market effect the other stock market in the same or different regions, then we can say that there is multivariate relationship existed between them. To find the relationship between volatilities and co-volatilities of several univariate stock markets then we can use the Multivariate GARCH model. DCC GARCH is a type of the Multivariate GARCH methodology. The motivation of using Multivariate methodology is to find the correlation between the volatility between two or more stock markets. Another motivation is to make the portfolio allocation on the basis of co-integrated markets and spillover impact. The volatility in one stock market transfers to the other stock market, it means that these markets are co-integrated. Investors are more critical for making investment in co-integrated markets. In this study, we used the DCC GARCH model because DCC GARCH model parametrized the conditional correlation directly. In view to DCC-GARCH, the one stock market interdependence on the other stock market. The relationship between two or more variables which depend on previous past information that changes over time, not constant, is the Dynamic condition correlation GARCH (DCC-GARCH) model. The conditional correlation in the DCC-GARCH model is measured by the two parameters DDC Alpha (γ1) and DCC Beta (γ2). Both γ1 and γ2 indicate the dynamic and time varying behavior in the model estimated. DDC Alpha (γ1) describes the short run volatility impact from one economy to another economy, which also indicates the persistency in the standard residual from previous period. DCC Beta (γ2) measures the lingering effect of the shock, which is persistent of conditional correlation in the model. The sum of these two parameters should be less than one that indicated the conditional correlation in the model are not constant over time and has dynamic behavior.

Similarly, if DDC Alpha (γ1) value is not significant, it means that there is not short-term persistence found between two stock market, where as the DCC Beta (γ2) shows the long-term persistence between the two stock markets. In our results in Table 4, pair Malaysia-France DDC Alpha (γ1) is significant, indicated the short-term spillover impact of Malaysian indices over France index. DCC Beta (γ2) also in this pair significant that indicated the long-term spillover impact of Malaysian index over France. From the Malaysia-France pair, we can conclude that there is dynamic relationship existed between two stock markets. Our results also shows that the volatility in the Malaysian stock market effect the volatility in stock market of France for both short and long period of time. Similarly, Malaysia- Germany, Malaysia- India, Malaysia-Japan, Malaysia- Pakistan, Malaysia-Singapore, Malaysia-UK, Malaysia-Indonesia and Malaysia-China pairs DDC Alpha (γ1) and DCC Beta (γ2) is significant, indicating the short- and long-term persistence in the volatility between Malaysia and other group pairs. Malaysian stock market indices have the short term and long-term spillover impact on all the selected countries except USA. In case of Malaysia-USA pair, the DDC Alpha (γ1) and DCC Beta (γ2) is not significant, it means that there is not dynamic relationship existed between these two stock markets. From our results, we can summarize that the volatility in the Malaysian market effected the other trading partners stock market for both short and long run and hence, we can say that risk co-movement transfer from Malaysia to its trading partners except USA.

**Table 4:** Results DCC-GARCH model.

Pair	DDC Alpha (γ1)	P-value	DCC Beta (γ2)	P-value
Malaysia-France	0.0139***	0.0000	0.9693***	0.0000
Malaysia- Germany	0.0124***	0.0004	0.9695***	0.0000
Malaysia- India	0.0131***	0.0000	0.9806***	0.0000
Malaysia-Japan	0.0125***	0.0022	0.9772***	0.0000
Malaysia- Pakistan	0.0100**	0.0252	0.9569***	0.0000
Malaysia-Singapore	0.0274***	0.0000	0.9584***	0.0000
Malaysia-UK	0.0142***	0.0001	0.9629***	0.0000
Malaysia- USA	-0.0051	0.2684	0.4602	0.5760
Malaysia-Indonesia	0.0160***	0.0000	0.9780***	0.0000
Malaysia-China	0.0071***	0.0000	1.0015***	0.0000

## 5. Concluding remarks and policy implication

We investigate in our study the causality relationships between the Malaysian stock market and its trading partners and the co-movement dynamic risk behavior. Using different wavelet techniques, we demonstrate different risk co-movements in the short and long run, as well as in both OECD and emerging markets. We conclude that the risk co-movement is sustainable in both the short and long run and in both OECD and emerging markets over time.

In recent years, research has focused mostly on the co-movements of risk among financial markets of the different regions, including developed, emerging, and less developed economies. The theoretical discussion can be broadly divided into two groups. The first group includes fundamentally based authors who claim that stock market co-movement is an inevitable result of trade connectivity movement. The second group of authors are non-fundamental authors dependent on non-fundamental causes for stock market interdependence. This study chooses Malaysia as a special case to study, referred to by the first category, to investigate the risk co-movement with its trading partners on the basis of various time-frequency frameworks. Our main hypothesis is that trading connectivity causes stock market integration, measured by co-movement patterns. Particularly, we aimed to answer these objectives: 1) What is the effect of risk and causality transmission from the Malaysian stock market to its trading partners before and after the crisis (means different tome-frequency domain)? It means we will find the risk co-movement and Causality between Malaysia and its trading partners from two different regions. We applied a detailed Wavelet to answer these research questions: Cross wavelet (XWT), wavelet Coherence (WCOH), and robustness through the wavelet Granger causality, and DCC-GARCH. Our empirical findings reveal significant evidence of risk co-movement between the Malaysian stock market and its trading partners during different frequency and time domains. More interestingly, Malaysia has a positive relationship with all selected emerging as well as the OECD stock market during the period of financial crisis and COVID-19. In addition, Malaysia is leading the stock market of India, USA, France, Germany, Japan, Pakistan, and the UK in the period of financial crisis 1997–98 in the low-frequency domain, which means that for the short run. In the period of the financial crisis of 1997–98, Malaysia is lagging behind China due to the larger interdependence between them. During the COVID-19 pandemic (2020–21), the Malaysian stock market was driven by two major trading partners, including Indonesia and China.

Furthermore, the Granger causality test shows the bi-directional and unidirectional causality between Malaysia and its trading partners over the four frequency domains. This is consistent with the idea that there will not be an issue of the leadership position between the Malaysian stock market and its trading partners in the long run, except for Indonesia, Singapore, and China. Our Granger causality findings imply that the temporary shocks of the developed or OECD country’s stock market directly impact the Malaysian stock market, extending to the longer scale. At the same time, proximity does not affect stock market correlation as Malaysia and its trading partners need longer to absorb each stock market shock and adjust their prices accordingly. In addition, our time-frequencies domains causality analysis (D1, D2, D3, and D4) sheds light on the time required by the Malaysian market to interact with its trading partners and the nature of the lead-lag relationship. This time-frequency is very helpful for the investors to decide the investment in Malaysian stock market by considering the shock effect and its captured period. Moreover, our DCC-GARCH findings shows that Malaysian market shows both short term and long term volatility pattern with trading partners except USA on the ground of the trade agreements and trade flow.

Overall, our study contributes to studies showing that the Malaysian stock market risk significantly affects other stock market risks, either in the Asian emerging region or OECD regions, emphasizing thus the substantial role Malaysia is playing in the rest of the world [69, 70]. Furthermore, our research demonstrates that interdependence between stock markets is substantially correlated with trade, economic integration, and economic relationships. For instance, it has been suggested by [53, 71] that trade flow between the economies is likely to be the driving force behind open regionalism in capital markets.

We also offer evidence to contradict claims made by certain researchers that stock market segmentation can coexist with regional trading blocks and international economic links, such as the ASEAN Free Trade Area [61] and the North American Free Trade Area (NAFTA) [72]. Additionally, we present evidence contradicting studies that claim Malaysia is cut off from developed Asian as well as OECD markets. However, since Malaysia joined the World Trade Organization in 1995, the relationship between the Malaysian stock market and the rest of the world changed. More recently, the ASEAN Trade in Goods Agreement (ATIGA), the Trans-Pacific Partnership Agreement (TPPA), the Comprehensive and Progressive Agreement for the Trans-Pacific Partnership (CPTPP), Malaysia-European Free Trade Area Economic Partnership Agreement (MEEPA), Malaysia-EU Free Trade Agreement (MEUFTA) and others trade agreements enforce its global leadership in term of trade and economic weight and also international financial integrations.

Given the significance of our study, we argue that our findings have some important and useful implications. We find the weak co-movement between Malaysia and Pakistan. Hence, these weak correlation countries are the best choice for Malaysian investors, and Pakistani investors have the best investment choice in Malaysia. In this way, they can diversify their portfolio. In addition, investors and fund managers are urged to modify their allocations in light of our time-frequency findings, considering the choice of countries and the length of the investment horizons, particularly how the stock markets in Malaysia and its trading partners react to regional or global shocks and crises. To adjust their fiscal and monetary policies, policymakers in these countries consider local and international shocks and be aware of the type and frequency of their stock market integration. This study contains some intriguing contributions regarding Malaysia’s stock market dependence on international stock markets. However, we were limited to stock market co-movement analyses. We propose controlling other driving elements in future studies. In addition, integrating additional trading partners would provide further insight into the relationship between trade connectedness and stock market integration.

Moreover, in line with improving the technical precision of the empirical findings, this study can be held using other techniques such as machine learning and others. Moreover, different economies of different economic types can be part of future research investigating the risk and causality transmission due to globalization. Future research should be conducted on the role of the government in maintaining the stock market, especially during crises and pandemics.

## Supporting information

S1 Data (XLSX)
